The article "Influence of Dexmedetomidine on Diaphragm Function and Postoperative Outcomes in ICU Patients with Mechanical Ventilation" was retracted in 2023. Reasons: unreliable results or conclusions; concerns about the data; concerns about the peer review; concerns about the citations.

# Influence of Dexmedetomidine on Diaphragm Function and Postoperative Outcomes in ICU Patients with Mechanical Ventilation

**DOI:** 10.1155/2021/1990838

**Published:** 2021-10-25

**Authors:** Chengda Zhao, Meihua Huang, Baiyun Wang, Huanhui Zhong, Wen Meng

**Affiliations:** ^1^The Affiliated Nanhua Hospital, Department of Anesthesiology, Hengyang Medical College, University of South China, Hengyang 421001, Hunan, China; ^2^Corporate Office, Drug Clinical Trial Center of Hengyang Huacheng Hospital, Hengyang 421001, Hunan, China; ^3^The Affiliated Nanhua Hospital, Department of Critical Care Medicine, Hengyang Medical College, University of South China, Hengyang 421001, Hunan, China

## Abstract

**Objective:**

To probe into the influence of dexmedetomidine (DEX) on diaphragm function and postoperative outcomes of mechanically ventilated patients in the intensive care unit (ICU).

**Methods:**

84 patients with mechanical ventilation (MV) in the ICU of our hospital were selected as the research participants, including 38 patients in the control group (CG) sedated with midazolam (MZ) and 46 patients in the research group (RG) with DEX sedation. Ramsay sedation score, visual analogue scale (VAS), and restlessness score (RS) were used to evaluate their state before sedation (T0), as well as 2 h (T1), 6 h (T2), and 24 h (T3) after sedation, and the alterations of mean arterial pressure (MAP) and heart rate (HR) were recorded. Serum cortisol (Cor), adrenocorticotropic hormone (ACTH), superoxide dismutase (SOD), malondialdehyde (MDA), interleukin- (IL-) 1*β*, IL-6, and tumor necrosis factor-*α* (TNF-*α*) were measured before and 24 h after sedation. The end-inspiratory diaphragm thickness (DTei) and end-expiratory diaphragm thickness (DTee) were measured within 2 h after the initiation of MV and 5 min after the spontaneous breathing test (SBT), and the diaphragm thickening fraction (DTF) was calculated. Finally, the ventilator weaning, MV time, and the incidence of adverse reactions (ADs) of the two groups were counted.

**Results:**

T0 and T3 witnessed no distinct difference in Ramsay, VAS, and RS scores between the two arms (*P* > 0.05), but at T1 and T2, RG had better sedation state and lower VAS and RS scores than CG (*P* < 0.05), with more stable vital signs (*P* < 0.05). After sedation, the contents of oxidative stress and inflammatory factors in RG were lower, while DTee, DTei, and DTF were higher, versus CG (*P* < 0.05). Moreover, RG presented higher success rate of first ventilator weaning, less MV time, and lower incidence of ADs than CG (*P* < 0.05).

**Conclusions:**

DEX is effective in mechanically ventilated patients in the ICU, which can protect patients against diaphragm function damage, improve the success rate of ventilator weaning, and benefit the postoperative outcome, with excellent and rapid sedation effect and less stress damage to patients.

The article "Influence of Dexmedetomidine on Diaphragm Function and Postoperative Outcomes in ICU Patients with Mechanical Ventilation" was retracted in 2023. Reasons: unreliable results or conclusions; concerns about the data; concerns about the peer review; concerns about the citations.

## 1. Introduction

Most of the patients transferred to the intensive care unit (ICU) are in critical condition, and these patients are usually accompanied by organ failure of different degrees, among which the most common manifestation is decreased and disordered respiratory function [1]. In order to ensure the life safety of patients, most patients in the ICU need to implement mechanical ventilation (MV) intervention, i.e., endotracheal intubation through the nose and mouth, to change the patient's spontaneous breathing movement through a ventilator to maintain airway patency [2]. The use of MV can effectively ensure the normal breathing of patients and prevent serious respiratory diseases caused by hypoxia injury and carbon dioxide accumulation [3]. However, the intense pain caused by MV greatly influences patients' treatment experience and compliance [4]. In addition, MV is accompanied by certain irritation and infectivity, which may further cause inflammatory injury, oxidative stress (OSR), and even infectious diseases in heart and lung tissue [5]. Moreover, due to various influences of MV and the disease itself, patients will experience varying degrees restlessness, resistance, and rebellious psychology during treatment, which seriously affects the efficiency of clinical treatment [6]. Therefore, for the ICU, which is the key department to save patients' lives, paying attention to the application of MV and improving patients' comfort while maintaining their breathing are of great significance to improve the postoperative outcome of patients.

In clinical practice, patients who receive MV are usually given corresponding sedative adjunctive treatment, and their restlessness is relieved by anesthesia and sedation, so that the treatment can be implemented better [7]. The commonly used sedatives are opioid receptor agonists (fentanyl, etc.), with excellent sedative effects. However, there are obvious respiratory depression, unstable hemodynamics, and other adverse conditions, and the postoperative prognosis of patients is generally poor [8]. Consequently, the clinic is looking for a sedative scheme with high safety that can effectively achieve sedative effects. With the deepening of the research, we found the increasing critical role of dexmedetomidine (DEX) in MV [9, 10]. As an *α*2-adrenoceptor agonist, DEX has excellent inhibitory action on sympathetic nerve activity and catecholamine release, contributing to stable hemodynamics [11]. DEX can be absorbed rapidly after subcutaneous injection, with a peak time of about 1 h, and can be excreted in urine after metabolism [12]. DEX, as a stable and safe sedative drug, is extensively applied in various clinical general anesthesia operations, and has gradually demonstrated its excellent effect in MV [13, 14]. However, we found that currently, the application of DEX and sedation of patients with MV are usually limited to monitoring the alteration of patients' real-time vital signs, while ignoring their postoperative outcomes. In addition, diaphragm, as the most important respiratory muscle of the body, bears 60%–80% of the ventilation needs. Diaphragmatic dysfunction (DD) is a common adverse reaction after sedation, and it is also one of the key factors leading to adverse outcomes after operation [15]. The related research on DEX and diaphragm function of patients is also relatively rare.

The article "Influence of Dexmedetomidine on Diaphragm Function and Postoperative Outcomes in ICU Patients with Mechanical Ventilation" was retracted in 2023. Reasons: unreliable results or conclusions; concerns about the data; concerns about the peer review; concerns about the citations.

At present, MV is a necessary measure to protect patients' lives, and finding a better sedation scheme is the key link to improving the treatment efficiency of patients. This study aims to further inquire into the application value of DEX in MV by exploring the impacts of DEX on the diaphragm function and postoperative outcomes of mechanically ventilated patients in the ICU, so as to provide more comprehensive and reliable reference and guidance for future clinical practice.

## 2. Materials and Methods

### 2.1. General Information

This prospective analysis included 84 patients with postoperative MV in the ICU of our hospital between May 2020 and June 2021, including 38 patients in the control group (CG) sedated with midazolam (MZ) and 46 patients in the research group (RG) with DEX sedation. This research was ratified by the hospital ethics committee, and all the enrolled participants provided the informed consent signed by themselves or their next of kin.

### 2.2. Eligibility Criteria

Inclusion criteria: (1) age ≥18 years; (2) nasal or orotracheal intubation, MV >48 h; (3) being admitted to the ICU for more than 24 h; and (4) normal cognitive function.

Exclusion criteria: (1) there are contraindications to sedatives such as MZ and DEX; (2) need long-term noninvasive ventilator support; (3) coma or confusion, neuromuscular disease, high paraplegia, multiple rib fractures, flail chest, airway obstruction, etc.; (4) mental illness; (5) long-term use of sedative and analgesic drugs; (6) major progress is made during the study; and (7) severe nervous system diseases, such as severe brain trauma, acute cerebral infarction, and acute intracranial hemorrhage.

### 2.3. Methods

Both groups received MV and fentanyl (Yichang Humanwell Pharmaceutical, SFDA Approval No. H20030197) for analgesia after admission to ICU. On this basis, CG was given 0.03–0.30 mg/kg MZ (Jiangsu Nhwa Pharmaceutical, SFDA Approval No. H1990027) for sedation intravenously, and the patient's sedation degree was observed to maintain sedation at 0.04–0.20 mg/kg/h. In RG, 0.5–1.0 *μ*g/kg DEX (Yangtze River Pharmaceutical Group, SFDA Approval No. H20183219) was injected intravenously and completed within 10–15 min, and the sedation was observed and maintained at 0.2–0.4 *μ*g/kg/h.

The article "Influence of Dexmedetomidine on Diaphragm Function and Postoperative Outcomes in ICU Patients with Mechanical Ventilation" was retracted in 2023. Reasons: unreliable results or conclusions; concerns about the data; concerns about the peer review; concerns about the citations.

### 2.4. Endpoints

1. Sedation: Ramsay sedation score was utilized to evaluate patients' sedation degree before sedation (T0), as well as 2 h (T1), 6 h (T2), and 24 h after sedation (T3). Grade I: the patient showed restlessness, anxiety, and irritability; grade II: the patient was stable and can obey the doctor's instructions; grade III: the patient had mild response to the doctor's instructions; and grade IV: the patient fell asleep deeply, with no response to stimulation.
2. Somatosensory status: patients' somatosensory status was assessed using visual analogue scale (VAS) and restlessness scale (RS). The higher the VAS and RS scores, the more obvious the pain and restlessness of patients.
3. Vital signs: the alterations of mean arterial pressure (MAP) and heart rate (HR) were recorded.
4. OSR: before and after 24 h after sedation, 4 milliliters of venous blood were sampled from patients into coagulation-promoting tubes, which were left at ambient temperature for 30 min and then centrifuged to obtain serum, for the determination of cortisol (Cor), adrenocorticotropic hormone (ACTH), superoxide dismutase (SOD), and malondialdehyde (MDA) by ELISA.
5. Inflammatory reaction: serum levels of interleukin- (IL-) 1*β*, IL-6, and tumor necrosis factor-*α* (TNF-*α*) were detected.
6. Diaphragm function: the ventilator was set to pressure support ventilation 24 h after the start of the spontaneous breathing test (SBT). The end-inspiratory diaphragm thickness (DTei) and end-expiratory diaphragm thickness (DTee) were measured within 2 h after MV and 5 min after SBT, and the diaphragm thickening fraction (DTF) = (DTei-DTee)/DTei × 100%.
7. Ventilator weaning: weaning was carried out in strict accordance with the MV guidelines of the American College of Chest Physicians (ACCP). If the patient did not need re-MV support within 48 h after weaning, it was considered as a successful weaning, while if SBT failed or intubation and MV was resumed 48 h after weaning, the weaning was deemed failed. The two arms were compared for the success of the first weaning, and the MV time was recorded.
8. Safety: adverse reactions (ADs) during MV in both arms were recorded, and the incidence of ADs was calculated.

The article "Influence of Dexmedetomidine on Diaphragm Function and Postoperative Outcomes in ICU Patients with Mechanical Ventilation" was retracted in 2023. Reasons: unreliable results or conclusions; concerns about the data; concerns about the peer review; concerns about the citations.

### 2.5. Statistical Processing

The experimental results were processed statistically by SPSS22.0 software. The success rate of the first weaning and AD incidence were expressed by percentages and analyzed by the chi-square test. Ramsay, VAS, and RS scores, AP and HR changes, Cor, ACTH, SOD, MDA, IL-1*β*, IL-6, and TNF-*α* levels, and DTei, DTee, and MV time, described as (mean ± standard deviation), were compared by the *T* test, one-way ANOVA, and LSD post hoc test. Significance was set at a *P* value of <0.05.

## 3. Experimental Results

### 3.1. Comparison of Baseline Data

As shown in Table 1, the clinical baseline data were not evidently different between the two arms (*P* > 0.05).

### 3.2. Comparison of Analgesic Effects

T0 and T3 witnessed no distinct difference in the Ramsay sedation score between the two arms (*P* > 0.05), but at T1 and T2, RG had better sedation state than CG (*P* < 0.05). In RG, only 2 patients achieved excessive sedation (grade V) at T3, compared with 6 patients in CG, as shown in Table 2.

### 3.3. Comparison of Somatosensory Status

As shown in Figure 1, VAS and RS scores at T0 and T3 in RG showed no difference compared with CG (*P* > 0.05), while the scores at T1 and T2 were lower versus CG (*P* < 0.05). In both arms, the VAS and RS scores of patients decreased gradually with the sedation time (*P* < 0.05).

### 3.4. Comparison of Vital Signs

As shown in Figure 2, MAP and HR differed insignificantly between the two arms at T0, T2, and T3 (*P* > 0.05), while they were lower in RG than in CG at T1 (*P* < 0.05). In RG, MAP and HR were similar at T1, T2, and T3, which were all lower than those at T0 (*P* < 0.05), while in CG, MAP and HR at T1 were lower than T0 and even lower at T2 (*P* < 0.05), and there was no difference between T3 and T2 (*P* > 0.05).

### 3.5. Comparison of OSR

As shown in Figure 3, Cor, ACTH, SOD, and MDA were similar in the two arms before sedation (*P* > 0.05); however, Cor, ACTH, and MDA decreased and SOD increased in both arms after sedation, and the alterations were more evident in RG (*P* < 0.05).

### 3.6. Comparison of Inflammatory Reactions

As shown in Figure 4, the contents of inflammatory factors (IFs) IL-1*β*, IL-6, and TNF-*α* of the two arms were not different before sedation (*P* > 0.05), whereas the abovementioned IFs dropped in both arms after sedation, especially in RG (*P* < 0.05).

### 3.7. Diaphragm Function

As shown in Figure 5, DTee, DTei, and DTF differed insignificantly between the two arms after MV (*P* > 0.05); after SBT, however, DTee, DTei, and DTF declined in both arms and were higher in RG (*P* < 0.05).

### 3.8. Comparison of Ventilator Weaning

As shown in Table 3, the success rate of the first weaning in RG was 95.65%, which was higher than that in CG (*P* < 0.05). In addition, none of the patients in RG while 2 in CG died after weaning. The MV time in RG was (5.25 ± 1.53) d, which was notably lower than that in CG (*P* < 0.05).

The article "Influence of Dexmedetomidine on Diaphragm Function and Postoperative Outcomes in ICU Patients with Mechanical Ventilation" was retracted in 2023. Reasons: unreliable results or conclusions; concerns about the data; concerns about the peer review; concerns about the citations.

### 3.9. Comparison of Safety

As shown in Table 4, the incidence of ADs was evidently lower in RG (4.35%) than in CG (18.42%) (*P* < 0.05).

### 3.10. Discussion

MV is a common way of respiratory support for critically ill patients in the ICU, with relevant data indicating that approximately 70% of ICU patients need MV [16]. However, due to the influence of many factors, MV will inevitably lead to adverse postoperative outcomes, such as weaning difficulties caused by serious respiratory fatigue, spontaneous respiratory arrest, and prolonged treatment time [17]. Referring to the previous data, we found that DD was one of the important reasons for the difficulty and failure of weaning [18]. Therefore, active prevention and treatment of DD is of great significance to help patients recover as soon as possible and improve postoperative outcomes. MZ and DEX, as common clinical anesthetics, have shown good effects in sedation during MV. However, their effects on diaphragm function and postoperative outcomes are rarely reported, and the comparison of clinical effects between them is still controversial. Therefore, this study is of great significance to the selection of clinical sedatives in the future by discussing and comparing their effects in ICU patients undergoing mechanical ventilation.

First, we compared patients' baseline data and found no difference, which confirmed the comparability between the two groups and guaranteed the accuracy of the experimental results. Then, we used Ramsay sedation score to evaluate sedation and found that there was no significant difference between the two groups after 24 hours of sedation, which indicated that DEX and MZ had stable and effective sedation effects. However, Ramsay scores were better in RG at 2 h and 6 h of sedation, which suggested that DEX could make patients enter a stable state more quickly. We also proved this when we used VAS and RS to evaluate patients. It is shown that patients with MV in the ICU are prone to emergence agitation during treatment, which can easily induce many adverse events and affect the treatment effect [19]. Our experimental results also further suggest that DEX has a good sedative effect, which can relieve the agitation of patients to a certain extent and improve the treatment compliance. We believe that this may be due to the pharmacological mechanism of DEX. Brainstem locus coeruleus is responsible for regulating sleep and awakening in the human brain, and *α*2 receptors are the most concentrated receptors in the central nervous system of this part, which can produce sleep-like analgesic, sedative, and antianxiety effects by acting on *α*2 adrenergic receptors in the spinal cord and brainstem locus coeruleus of patients [20]. Different from traditional medicine MZ, DEX has a sedative effect on patients outside the cerebral cortex and can produce a sedative effect similar to that of normal sleep [21]. Besides, as an *α*2-adrenoceptor agonist, DEX has a high affinity with *α*2, and *α*2 receptors are mainly distributed in the presynaptic membrane and can inhibit the release of norepinephrine and the activity of neurons [22]. Also, via activating presynaptic membrane *α*2 receptors, DEX can inhibit the transmission of pain signals and reduce pain to achieve anesthesia. Additionally, DEX can suppress the activity of sympathetic nerves by activating postsynaptic membrane *α*2 receptors, causing a series of sedative effects such as lowering blood pressure and heart rate, thus stabilizing the hemodynamics of patients and the normal activities of the heart and achieving the protection of heart and myocardial tissue [23]. When investigating patients' vital signs, we found that, after the application of DEX, the patients quickly entered a stable state, without obvious alterations in their MAP and HR. On the other hand, although MZ also has a stable effect, its effectiveness is obviously not as good as DEX. In addition, we found in previous studies that DEX can inhibit sympathetic nerve excitement and reduce stress response of the body [24]. Hypothalamic-pituitary-adrenal (HPA) axis is the main pathway used by the body to regulate stress response. When the body is stimulated by stress, HPA will be activated, and the synthesis and secretion of ACTH will increase, thus inducing a large amount of secretion of Cor and increasing its expression in the body [25]. After sedation, ACTH, Cor, and oxidative metabolite MDA decreased, while SOD increased, indicating the excellent application effect of DEX in MV, which was of great significance to prevent intubation infection and inflammatory injury in patients. Moreover, the levels of IFs in patients were evidently suppressed, which can prove our point of view.

The article "Influence of Dexmedetomidine on Diaphragm Function and Postoperative Outcomes in ICU Patients with Mechanical Ventilation" was retracted in 2023. Reasons: unreliable results or conclusions; concerns about the data; concerns about the peer review; concerns about the citations.

The diaphragm is the most important inspiratory muscle in respiratory muscles, and DD, one of the serious complications faced by ICU patients with MV, will lead to the impairment of normal ventilation function [26]. By testing patients' diaphragm function, we found that, after SBT, the DTee, DTei, and DTF decreased in both arms, with obvious higher parameters in RG. It suggests that the diaphragm function of the two groups is damaged to varying degrees after MV, but the application of DEX can make the diaphragm function of the patients less damaged. DD, as a key factor affecting respiratory depression, is also a key link to determine the success rate of weaning to a great extent. As expected, the success rate of weaning was naturally increased as the patients in RG had less damage to diaphragm function. Finally, we compared the safety between the two arms and found a lower incidence of ADs in RG. It reconfirms the safety of DEX in MV, which is also consistent with the previous studies [21, 26].

However, due to limited experimental conditions, there are still some shortcomings to be addressed in this study. For example, the research cycle is too short to clarify patients' long-term prognosis. Besides, there are many kinds of sedative drugs used in clinics, so we need to compare DEX with other drugs to improve the comprehensiveness of our results. Moreover, due to the lack of basic experiments, we cannot determine the exact mechanism of DEX on patients. We will conduct a more complete experimental analysis on the abovementioned deficiencies as soon as possible to obtain more effective experimental results for clinical reference.

## 4. Conclusions

Collectively, DEX is effective in ICU MV, which can protect patients against diaphragm function damage, improve the success rate of weaning, and facilitate patients' postoperative outcomes, with excellent and rapid sedation as well as less stress damage to patients.

## Figures and Tables

**Figure 1:** Comparison of somatosensory status. (a) VAS scores. (b) RS scores. ^*∗*^: vs. RG, *P* < 0.05. ^#^: vs. T0, *P* < 0.05. &: vs. T1, *P* < 0.05. @: vs. T2, *P* < 0.05.

**Figure 2:** Comparison of vital signs. (a) MAP. (b) HR. ^*∗*^: vs. RG, *P* < 0.05. ^#^: vs. T0, *P* < 0.05. &: vs. T1, *P* < 0.05.

**Figure 3:** Comparison of oxidative stress response. (a) Cor. (b) ACTH. (c) SOD. (d) MDA. ^*∗*^: vs. RG, *P* < 0.05. ^#^: vs. before sedation, *P* < 0.05.

**Figure 4:** Comparison of inflammatory reactions. (a) IL-1*β*. (b) IL-6. (c) TNF-*α*. ^*∗*^: vs. RG, *P* < 0.05. ^#^: vs. before sedation, *P* < 0.05.

**Figure 5:** Comparison of diaphragm function. (a) DTee. (b) DTei. (c) DTF. ^*∗*^: vs. RG, *P* < 0.05. ^#^: vs. before sedation, *P* < 0.05.

**Table 1:** Baseline data of patients.

Group	RG (*n* = 46)	CG (*n* = 38)	*t* or *χ*^2^	*P*
Age	65.5 ± 5.4	66.8 ± 5.6	1.080	0.283
Gender			0.752	0.386
Male	32 (69.57%)	23 (60.53%)		
Female	14 (30.43%)	15 (39.47%)		
Smoking			0.769	0.381
Yes	25 (54.35%)	17 (44.74%)		
No	21 (45.65%)	21 (55.26%)		
RCT (ng/mL)	18.72 ± 10.12	19.13 ± 9.45	0.565	0.573
BMI (kg/m^2^)	24.89 ± 3.34	24.48 ± 3.27	0.492	0.625
APACHE II score	24.43 ± 2.76	25.07 ± 2.81	1.049	0.297
Nationality			0.010	0.920
Han	31 (67.39%)	26 (68.42%)		
Minority	15 (32.61%)	12 (31.58%)		

The article "Influence of Dexmedetomidine on Diaphragm Function and Postoperative Outcomes in ICU Patients with Mechanical Ventilation" was retracted in 2023. Reasons: unreliable results or conclusions; concerns about the data; concerns about the peer review; concerns about the citations.

**Table 2:** Comparison of sedative effects.

Group	RG (*n* = 46)	CG (*n* = 38)	*χ* ^2^	*P*
T0			0.637	0.425
I/II/III/IV/V	46/0/0/0/0	37/1/0/0/0		
T1			6.108	0.047
I/II/III/IV/V	22/21/3/0/0	26/10/0/0/0		
T2			20.110	<0.001
I/II/III/IV/V	1/6/15/24/0	5/12/16/3/0		
T3			4.632	0.201
I/II/III/IV/V	0/4/6/38/2	0/2/2/28/6		

**Table 3:** Comparison of ventilator weaning.

Group	RG (*n* = 46)	CG (*n* = 38)	*χ* ^2^/*t*	*P*
The success rate of removing the ventilator	44 (95.65%)	28 (73.68%)	8.201	0.004
Mortality after removal of the ventilator	0 (0.00%)	2 (5.26%)	2.480	0.115
Mechanical ventilation time (d)	5.25 ± 1.53	6.71 ± 2.01	3.778	<0.001

**Table 4:** Incidence of adverse reactions.

Group	RG (*n* = 46)	CG (*n* = 38)	*χ* ^2^	*P*
Restlessness	1 (2.17%)	2 (5.26%)		
Respiratory depression	0 (0.00%)	2 (5.26%)		
Unstable blood pressure	1 (2.17%)	1 (2.63%)		
Delirium	0 (0.00%)	2 (5.26%)		
Total incidence	4.34%	18.41%	4.308	0.038

## Data Availability

The data are available from the corresponding author.
